The article "Integrating mechanisms of response and resistance against the tubulin binding agent Eribulin in preclinical models of osteosarcoma" was retracted in 2024. Reasons: fabricated or falsified data; errors in the data; errors in the text.

# Integrating mechanisms of response and resistance against the tubulin binding agent Eribulin in preclinical models of osteosarcoma

**DOI:** 10.18632/oncotarget.13358

**Published:** 2016-11-15

**Authors:** Valerie B. Sampson, Nancy S. Vetter, Wendong Zhang, Pratima U. Patil, Robert W. Mason, Erika George, Richard Gorlick, Edward A. Kolb

**Affiliations:** ^1^ Cancer Therapeutics Laboratory, Nemours Center for Cancer and Blood Disorders, Nemours/A.I. duPont Hospital for Children, Wilmington, DE, USA; ^2^ Department of Pediatrics - Hematology and Oncology, The Children's Hospital at Montefiore, The Albert Einstein College of Medicine, Bronx, NY, USA; ^3^ Nemours Center for Childhood Cancer Research, Alfred I. duPont Hospital for Children, Wilmington, DE, USA; ^4^ Department of Biological Sciences, University of Delaware, Newark, DE, USA

**Keywords:** eribulin, microtubule destabilization, G2/M arrest, mitotic catastrophe, cell death

## Abstract

Osteosarcoma is the most frequently occurring bone cancer in children and adolescents. Unfortunately, treatment failures are common. Eribulin is a synthetic microtubule inhibitor that has demonstrated activity in preclinical osteosarcoma models. The effects of eribulin were evaluated in two human osteosarcoma cell lines as well as in eribulin-sensitive and -resistant osteosarcoma xenograft tumors of the Pediatric Preclinical Testing Program (PPTP) by characterizing cell viability, microtubule destabilization, mitotic arrest and mechanism of cell death. Eribulin demonstrated cytotoxic activity *in vitro*, through promotion of microtubule dynamic instability, arrest of cells in the G2/M phase, mitotic catastrophe and cell death. The microtubule-destabilizing protein stathmin-1 (STMN1) was coimmunoprecipitated with the cyclin-dependent kinase inhibitor p27 indicating that these cytoplasmic complexes can protect cells from the microtubule destabilizing effect of eribulin. Increased tumoral expression of P-glycoprotein (P-gp) and *TUBB3* were also associated with lower drug sensitivity. In summary, eribulin successfully blocked cells in G2/M phase but interfered with mitochondria activity to inhibit proteins involved in apoptosis. Understanding the complex and inter-related mechanisms involved in the overall drug response to eribulin may help in the design of therapeutic strategies that enhance drug activity and improve benefits of eribulin in pediatric patients with osteosarcoma.

## INTRODUCTION

Osteosarcoma is the most frequent primary bone sarcoma that typically occurs in children and adolescents between 10 - 20 years of age [1]. Current multimodal therapy consisting of surgery with pre- and post–operative chemotherapy, achieves a 5-year survival rate of approximately 60 - 70% for non-metastatic high grade osteosarcoma patients [2, 3], while patients who present with metastatic disease at diagnosis have a 10 - 30% survival rate [4]. Chemotherapy agents that demonstrate anti-tumor activity in osteosarcoma include cisplatin, doxorubicin, ifosfamide and high dose-methotrexate [5]. Few other agents have shown efficacy. Consequently, treatment of existing metastatic disease and prevention of metastatic spread remain among the top challenges to increase long-term survival of patients. New therapeutic approaches and treatment strategies are being investigated to improve outcomes for patients with cancers that are resistant to current therapy.

Microtubules are dynamic structural cellular components. In proliferating cells, they are essential components in cell division through the formation of the mitotic spindle. Microtubule-targeting agents are generally classified as microtubule-stabilizers or microtubule-destabilizers. Destabilizing agents bind tubulin dimers and can inhibit tubulin polymerization (e.g. vinblastine) or drive polymerization (e.g. paclitaxel) causing suppression of microtubule dynamics that is essential for progression through mitosis [6]. Other microtubule-inhibitors bind tubulin polymers and stabilize microtubules and reduce the dynamics necessary for cell movement and division (e.g. taxanes and epothilones) or depolymerize microtubules and inhibit microtubule growth (e.g. vinca alkaloids). All of these agents lead to cell cycle arrest and can subsequently promote apoptosis, resulting in their clinical use as anti-cancer agents in the treatment of advanced breast and lung cancer. Microtubule-destabilizing agents (mainly vincristine) are currently used to treat some childhood cancers, while the microtubule-stabilizing taxanes are still in development.

Eribulin mesylate (eribulin, Halaven, Eisai Inc.) is a fully synthetic analogue of the natural marine sponge product halichondrin B, a macrocyclic ketone that targets microtubule dynamics [7]. It specifically binds with high affinity to the plus ends of microtubules, forming short, non-functional tubulin aggregates that suppress microtubule dynamic stability and inhibit microtubule growth [8]. This causes mitotic arrest by disrupting formation of normal mitotic spindles and subsequently leads to apoptosis of breast cancer cells [9]. Eribulin is currently approved for the treatment of recurrent metastatic breast cancer and improves overall survival in patients with late-stage metastatic disease [10]. In preclinical tests conducted by the Pediatric Preclinical Testing Program (PPTP), eribulin was well-tolerated in single-schedule studies and demonstrated potent activity in several childhood cancer models including osteosarcoma xenografts that were identified as either sensitive or resistant to drug [11]. Sensitive tumors demonstrated a statistically significant improvement in event-free survival (EFS) in the setting of a complete response, a partial response, stable disease, or progressive disease as defined previously [12]. Resistant tumors showed progressive disease and no improvement in EFS. Of the 6 xenograft tumors that were tested, 4 were eribulin-sensitive (OS1, OS2, OS17 and OS33), while 2 tumors were eribulin-resistant (OS9 and OS31) [11]. This pattern is consistent across other microtubule targeted therapies evaluated by the PPTP including paclitaxel [13], cabazitaxel and docetaxel [14].

Clinical trials to test the safety and efficacy of eribulin in pediatric patients are completed or underway: NCT02171260 is a Phase 1 study in patients with recurrent or refractory solid tumors (excluding CNS but including lymphomas) and NCT02082626 is a Phase 1 trial for children with cancer with no curative treatment options. The Children's Oncology Group (COG) recently completed a single-arm Phase II study of eribulin for recurrent osteosarcoma (AOST1322, NCT02097238) that failed to demonstrate any clinical responses [15].

Although microtubule-targeting drugs have been used extensively for cancer treatment in recent years, limitations include neurological and bone marrow toxicity and development of drug resistance. A better understanding of specific biological responses to microtubule-binding agents is critical for the development of novel therapeutic strategies. It is well-established that inhibition of microtubule spindle dynamics can affect various regulatory proteins and functions of cell organelles, including the Golgi apparatus, the endoplasmic reticulum, lysosomes and mitochondria [16]. Therefore, disruption of intracellular trafficking could provide an alternative drug-related toxicity during treatment with microtubule-targeting drugs. Among processes associated with resistance to microtubule-targeting drugs are mutations in β-tubulin or p53, expression of P-glycoprotein (P-gp), overexpression of βIII-tubulin or microtubule-interacting proteins (e.g. stathmin-1, STMN1) or microtubule-association proteins (MAPs) [reviewed in [17]]. More recently, gene signatures associated with transitions in cellular differentiation between epithelial and mesenchymal states are being studied as predictive biomarkers in osteosarcoma [18]. Apoptosis is commonly regarded as the major mechanism of cell death induced by eribulin [8], but other studies show that defects in the apoptotic default pathway downstream of microtubule insults can cause variations in the apoptotic response [19] or lead to necrosis [20]. The significance of these alternative pathways for prognosis or clinical value for pediatric cancers is not known.

The primary goal of this study is to identify molecular pathways affected by microtubule inhibition in preclinical cellular models that may determine drug efficacy in clinical trials. We used two osteosarcoma cell lines with different p53 status and metastatic properties and the PPTP osteosarcoma xenograft tumor panel to study effects of eribulin on microtubule structure, mitotic cell cycle blockade, mitochondria activity and mechanisms of cell death. We evaluated the gene and protein expression of STMN1 and the cyclin-dependent kinase (CDK) inhibitor p27(Kip1), which are involved in microtubule dynamics and implicated in resistance to microtubule targeting agents. Additionally, we examined the relationship between these factors and the traditional clinicopathological risk factors P-gp, βIII-tubulin and activation of cell proliferation pathways in cellular responses to eribulin. These results demonstrate that several complex and inter-related processes result in sensitivity to eribulin, and identify biomarkers that may have prognostic value in identifying pediatric patients with osteosarcoma who may respond favorably to eribulin.

## RESULTS

### Osteosarcoma cell lines demonstrate high sensitivity to eribulin

We examined the effects of eribulin on the proliferation of two osteosarcoma cell lines, SaOS and 143B. Cells were treated with 0.01 nM to 1000 nM eribulin for 72 hours and quantities of viable cells were compared to untreated samples using the cell titer blue assay. The IC50 value for SaOS cells was 3.5 nM and for 143B cells, 8.0 nM, Figure 1A and 1B. The IC50 values were similar to those for another pediatric osteosarcoma cell line [21]. Although eribulin exhibited potent activity at low concentrations, a small percentage of cells (∼15% for SaOS and ∼5% for 143B) remained viable, even at high drug concentrations (500 – 1000 nM). Phase-contrast images illustrate that live cells treated with eribulin are morphologically indistinguishable from untreated cells (Figure 1C, 143B). This suggests that a subset of cells may escape drug toxicity. To explore this further, SaOS and 143B cells were initially treated with 10 nM eribulin for 72 hours, followed by treatment with either 10 nM or 1 nM eribulin for an additional 72 hours. Cell viability was measured 144 hours after the start of the experiment. Continuous culture for 144 hours in 10 nM eribulin resulted in 32% viable cells for SaOS and 38% for 143B, compared with untreated cells (Figure 1D). The percentage of viable cells in the 10/1 nM group was 37% for SaOS (p=0.09) and 51% for 143B (p<0.05), Figure 1E). This experiment demonstrated that some cells survived after continuous eribulin exposure. These cells regained proliferative potential and grew to a confluent monolayer once eribulin was removed (Supplementary Figure S1). To determine whether surviving cells represented a sub-population of cells with innate resistance to eribulin, viable SaOS and 143B cells following initial eribulin treatment were cultured in drug-free medium and the IC50 values for these cells were determined. The IC50 was 5.0 nM for the surviving SaOS (data not shown) and 9.0 nM for the surviving 143B cells (Figure 1F). These IC50s were similar to values for cells that were not previously treated (Figure 1A and 1B) indicating the cells surviving initial eribulin treatment remain sensitive to drug.

**Figure 1:** Treatment of human osteosarcoma cells with eribulin **A**. SaOS and **B**. 143B cells were treated with eribulin at given concentrations for 72 hours. Viable cells were measured using the cell titer blue assay. Data are presented as mean absorbance ±SE of six replicates, n = 6. **C**. Representative phase-contrast images of live 143B cells that were treated with 10 nM eribulin for 72 hours. Scale bar - 200 μm. Arrows show live cells. **D**. Two groups of SaOS and **E**. two groups of 143B cells were treated with 10 nM eribulin for 72 hours, then one group was given 10 nM eribulin for an additional 72 hours (10_144h) and the other 1 nM eribulin for an additional 72 hours (10_72h/1_72h). Viable cells were measured using cell titer blue assay. Data are mean absorbance ±SE, n = 6. Asterisks denote statistically significant differences for the two treatment groups, *p< 0.05. **F**. 143B cells were treated with 10 nM eribulin for 72 hours. Surviving cells were cultured in drug-free media for 5 days then cells were treated with eribulin at given concentrations for 72 hours and cell viability was assessed. Data are presented as mean absorbance ±SE of six replicates, n = 6. **G**. Immunoblot analysis was performed on lysates of SaOS and 143B cells either untreated, treated with eribulin or subjected to drug washout (w/o) using antibodies against p-STAT3 (Y705), STAT3, p-Akt (S473), Akt, p42/44-MAPK and MAPK. GAPDH was loading control.

We also evaluated the effect of eribulin on proliferative and survival pathways. Signaling through the MAPK and STAT3 pathways promotes osteosarcoma cell proliferation and survival, while signaling through the Akt pathway regulates cell growth and apoptosis [22]. Immunoblot analysis demonstrated decreased total STAT3 and p-STAT3 levels in SaOS cells after 48 hours of exposure to 10 nM eribulin. Akt phosphorylation was lower in both cell lines after treatment, but a slight induction in p-MAPK was evident (Figure 1G). Reduced phosphorylation of STAT3 and Akt in treated cells is consistent with cytotoxicity while increased phosphorylation after drug washout is consistent with cell survival. STAT3 overexpression and activation is associated with poor prognosis in osteosarcoma. While eribulin reversibly blocked activation of STAT3 and Akt but not MAPK in SaOS cells, this effect was less pronounced in 143B cells, indicating that mechanisms of inhibition of cell proliferation were probably not the same in the two cell lines.

### Eribulin disrupts the microtubule network and triggers mitotic blockade in osteosarcoma cell lines

Tubulin-binding drugs disrupt normal mitotic spindle formation which can cause cell cycle arrest in mitosis and ultimately, cell death. We investigated the effect of eribulin on cellular tubulin and microtubule dynamics in SaOS and 143B by immunofluorescence and confocal microscopy. Cells were treated with 10 nM eribulin for 24 hours and immunolabelled using an anti-β-tubulin antibody. Immunofluorescence imaging showed that eribulin caused the formation of tubulin aggregates after 24 hours (Figure 2A – SaOS, panels i-vi and 143B, panels vii-xii). We assessed the effect of eribulin on cell cycle progression of SaOS and 143B cells by flow cytometric analysis after staining with propidium iodide. Representative cell cycle distribution plots are shown for 143B cells, Figure 2B. There was an increase in the percentage of SaOS and 143B cells in G2/M phase (Table 1) in response to eribulin compared to untreated cells. This demonstrates treatments led to cell cycle arrest in G2/M. We also evaluated the effect on expression of the cell cycle checkpoint protein cyclin B1 that is transiently expressed in the G2/M phase. Accumulation of cyclin B1 in G2/M is a known marker of cell cycle arrest [23]. Immunoblot of lysates of SaOS and 143B cells treated with eribulin for 48 hours showed increases in cyclin B1 expression compared to untreated controls (Figure 2C). When the drug is removed, cyclin B1 levels decreased, indicating that cells exit mitotic arrest to allow cell cycle progression and proliferation. Total levels of β-tubulin were unaffected by eribulin treatment (Figure 2C). We also assessed the response on the 6 PPTP osteosarcoma xenograft tumors [11] that were harvested from mice treated with eribulin for 48 hours. Immunoblot analysis showed there was marked upregulation in cyclin B1 protein in 5 treated xenograft tumors in comparison to control tumors (Figure 2D). Surprisingly, the OS9 tumor that is resistant to eribulin [11] has high expression of cyclin B1 with or without treatment. As seen for the cell lines, total levels of β-tubulin were unaffected by treatment (Figure 2D). Together, these results confirm that eribulin increases cyclin B1 expression which can lead to mitotic blockade in human osteosarcoma cell lines and xenografts, and that over-expression of cyclin B1 may be one of the factors that predicts sensitivity to therapy.

**Figure 2:** Microtubule disruption and β-tubulin aggregate accumulation induce expression of cell cycle regulators in osteosarcoma cell lines and xenograft tumors **A**. Confocal immunofluorescence imaging of β-tubulin (green) was performed on untreated SaOS (i – iii) and eribulin-treated SaOS (iv – vi) cells exposed to 10 nM eribulin for 24 hours. Panels vii – ix and x - xii show untreated and eribulin-treated 143B cells. Hoechst staining (blue) represent nuclei. Scale bars - 10 μm. **B**. 143B cells were either untreated or incubated with 10 nM eribulin for 24 hours and the cell cycle distribution was assessed by PI staining and flow cytometry analysis **C**. Immunoblot analysis was performed on lysates of SaOS and 143B cells that were either untreated, treated with eribulin or subjected to drug washout (w/o) using antibodies against cyclin B1 and β-tubulin. GAPDH was loading control. **D**. Untreated control osteosarcoma xenograft tumors and tumors harvested from mice treated with eribulin for 48 hours were lysed and assessed by immunoblot using antibodies against cyclin B1 and β-tubulin. GAPDH was loading control. **E**. Confocal immunofluorescence imaging of β-tubulin (green) and phase contrast imaging was done in eribulin-treated 143B cells that were regrown and treated with 10 nM eribulin for 24 hours. Hoechst staining (blue) represents nuclei. Scale bars – 7.5 μm.

**Table 1:** Effect of eribulin on the cell cycle distribution in SaOS and 143B osteosarcoma cell lines

	% of cells		
	G0/G1	S	G2/M
**SaOSUntreated**	39.94	23.71	21.32
**SaOSEribulin**	27.25	11.38	49.61
**143BUntreated**	28.94	23.77	18.39
**143BEribulin**	18.25	11.38	31.61

We also examined the effects of eribulin on the microtubule networks of surviving cells after initial treatment. Proliferating SaOS and 143B cells that were exposed to 10 nM eribulin for 72 hours were cultured in drug-free medium, and then incubated with or without 10 nM eribulin. After 24 hours cells were immunostained with anti-β-tubulin and examined by confocal microscopy (Figure 2E, panels i-iii). An intact microtubule network was observed in proliferating cells following drug washout, and these microtubule structures were disrupted in response to eribulin treatment (Figure 2E, panels iv-vi) indicating that surviving cells were sensitive to drug. These results suggest that heterogeneous populations of actively dividing and quiescent cells [24] could require either more drug or longer treatment regimens to be effective.

### Eribulin promotes non-apoptotic cell death in osteosarcoma cell lines and xenograft tumors

Immunofluorescence and phase-contrast images of 143B cells treated with eribulin for 48 hours (Figure 3A) show large, micronucleated cells with uncondensed chromatin (solid arrow) demonstrating that the drug induces mitotic catastrophe in osteosarcoma cells. Interestingly, a normal sized nucleus with condensed chromatin was observed in the adjacent cell (dotted arrow), indicating the responses to treatment were heterogeneous among cells. The nuclear morphology of a population of 143B cells treated with eribulin was analyzed by fluorescence microscopy (Figure 3B). Cells undergoing mitotic catastrophe were characterized by the appearance of enlarged multinucleated cells, aberrant nuclei clusters and decondensed chromatin. Approximately 70% of cells showed abnormal nuclei, illustrating mitotic catastrophe was induced in osteosarcoma cells (Figure 3B). The immunoblot in Figure 3C shows that levels of the histone *γ*-H2AX (and phosphorylation of ataxia telangiectasia mutated, ATM, data not shown) were unaffected by drug treatment in SaOS and 143B cells, suggesting that cells were devoid of direct DNA damage. These results demonstrate that treatment of osteosarcoma cells with eribulin promotes abnormal nuclei formation but not chromatin fragmentation.

**Figure 3:** Eribulin-induced mitotic catastrophe and necrosis in osteosarcoma cells **A**. Confocal immunofluorescence and phase contrast imaging was done on 143B cells treated with eribulin (10 nM) for 24 hours, then stained with Hoechst (blue) to visualize chromatin and with anti-β-tubulin antibody (green). Panel i, blue staining represents micronucleated chromatin (solid white arrow) and a single nucleus (dotted white arrow), panel ii represents cells visualized by phase contrast, panel iii represents β-tubulin (green), panel iv represents merged images. **B**. 143B cells were untreated (i) or treated with eribulin for 24 hours (ii) and nuclear morphology was evaluated using Hoechst staining (blue). Solid white arrows show abnormal nuclei, dotted arrows show normal nuclei. The percentage of cells containing normal and abnormal nuclei (mitotic catastrophe, mc) are expressed as mean ± SEM, n = 30 in each group. **C**. Immunoblot of lysates of SaOS and 143B cells either untreated, treated with eribulin, or subjected to drug washout (W/O), was performed using antibodies against PARP, cleaved PARP, caspase-3, Bcl-2, and *γ*-H2AX. GAPDH was loading control. **D**. Mitochondrial membrane potential was assayed by flow cytometry. Relative uptake of the cationic dye TMRE by SaOS and 143B cells is shown following 30 min and 24 hour eribulin treatments. Data are mean absorbance ±SE, for triplicate measurements. Asterisks denote statistically significant differences between untreated and treated cells, *p< 0.05. **E**. Untreated control osteosarcoma xenograft tumors and tumors harvested from mice treated with eribulin for 48 hours were lysed and assessed by immunoblot using antibodies against caspase-3 and Bcl-2. GAPDH was loading control.

We next investigated whether mitotic catastrophe culminated in apoptosis. Biochemical correlates of apoptosis (cleaved caspase-3, cleaved PARP and Bcl-2) were not elevated in eribulin-treated cells, Figure 3C. Since mitochondrial membrane damage induces apoptotic signal transduction, we assessed whether disruption of the microtubule network by eribulin affected the mitochondrial potential (ΔΨm). SaOS and 143B cells treated with eribulin, were subjected to the Mitochondrial Membrane Potential Assay and TMRE staining and analyzed by flow cytometry. In untreated 143B cells, TMRE accumulation in intact mitochondria of untreated cells resulted in high fluorescence, Supplementary Figure S2 and Figure 3D. In cells treated with eribulin a sub-population of cells with lower fluorescence intensity (panel iii, arrow) was detected after 30 min, indicating there was transient disruption of mitochondrial membrane potential. However, after 24 hours, only cells with high fluorescence were present (Figure 3D), indicating there was no loss of mitochondrial membrane potential which would allow these cells to enter apoptosis. Co-treatment with the mitochondrial protector olesoximine did not provide added benefits to the effects of eribulin (Supplementary Figure S2, panel v). Eribulin did not increase levels of cleaved caspase-3 in any of the xenograft tumors, confirming that apoptosis is not the mechanism of cell death in treated tumors [11], Figure 3E. Although Bcl-2 was expressed in 3 xenografts, OS1, OS2 and OS31, levels were not increased in response to drug treatment and expression was unrelated to drug sensitivity, Figure 3E. It is possible that necrotic cell death mediated by the kinase RIP1, and autophagy mediated by the upregulation of LC3 I/II occurred, Supplementary Figure S3. Taken together, our data suggest that eribulin treatment causes mitotic catastrophe but does not lead to apoptosis, and that cell death is most likely due to necrosis and/or autophagy.

### Accumulation of STMN1/p27 complexes protects osteosarcoma cells from the cytotoxic effects of eribulin

Several studies show that disruption of microtubules interferes with the intracellular transport of critical regulatory proteins [25]. The microtubule-sequestering protein STMN1 forms stathmin/tubulin complexes during the cell cycle and promotes microtubule depolymerization [26]. STMN1 is overexpressed in some osteosarcoma cell lines and its down-regulation increases sensitivity to taxanes [27]. The protein is located in the cytoplasm of SaOS cells (Figure 4A). We measured *STMN1* mRNA levels in cell lines and xenografts by real time RT-PCR and normalized values to HFL1 fibroblasts. As shown in Figure 4B, STMN1 was highly expressed in OS1, OS2, OS9 and OS33 tumors and lower in OS17 and OS31 relative to HFL1, but levels do not correlate with patterns of drug sensitivity. The protein p27 interacts with STMN1 to form STMN1/p27 complexes that do not bind β-tubulin, thereby preventing the role of STMN1 in microtubule destabilization [28, 29]. Immunoblot analysis showed eribulin treatment attenuated expression of both STMN1 and p27 in SaOS cells but in 143B cells only STMN1 protein decreased, and p27 levels slightly increased in response to eribulin, Figure 4C. We confirmed that p27 and STMN1 form complexes by immunoprecipitation from untreated and treated SaOS and 143B cells. Both proteins were detected in treated and untreated cells (Figure 4D). In the xenograft tumors, STMN1 protein increased in the eribulin sensitive tumors (OS9 and OS31) and one of the insensitive tumors (OS33). By contrast, p27 was only induced in the resistant tumors, OS9 and OS31 and not in the sensitive OS33 tumors (Figure 4E). We confirmed that p27 and STMN1 form complexes by coimmunoprecipitation experiments, Figure 4F. To determine the role of complexes in the sensitivity of osteosarcoma cells to eribulin, STMN1/p27 complex formation was disrupted by the knockdown of STMN1 using siRNA oligonucleotides targeting STMN1 in SaOS and 143B cells. Cell viability was measured following eribulin exposure at 2.5 nM for 48 hours. The cell viability data presented in Figure 4G and 4H demonstrate that SaOS and 143B cells treated with siRNA targeting STMN1 expressed reduced levels of STMN1 protein and were more sensitive to eribulin (11.5% viable cells) compared to cells that were treated with control siRNA and eribulin (36. 6% viable cells, p<0.05), Figure 4G and 4H. Taken together, we suggest that increased expression of both STMN1 and p27 in response to eribulin in resistant tumors increases accumulation of STMN1/p27 complexes and protects cells from the microtubule destabilizing effect of eribulin.

**Figure 4:** STMN1 expression and association with p27 **A**. Confocal immunofluorescence imaging of STMN1 (green) was performed on untreated SaOS (i – iii) and eribulin-treated SaOS (iv – vi) cells exposed to 10 nM eribulin for 24 hours. Panels vii – ix and x - xii show untreated and eribulin-treated 143B cells. Hoechst staining (blue) represent nuclei. Scale bars - 10 μm. **B**. Quantitative RT-PCR of STMN1 mRNA derived from each osteosarcoma xenograft tumor, shown as –fold change relative to HFL1. **C**. Immunoblot of lysates of SaOS and 143B cells untreated, treated with eribulin or subjected to drug washout (W/O) was performed using antibodies against p27 and STMN1. GAPDH was loading control. **D**. Lysates of SaOS and 143B cells either untreated or treated with eribulin were incubated with anti-STMN1 antibody. Immunoblots of immunoprecipitated complexes were probed with antibodies against STMN1 and p27. The extent of coimmunoprecipitation was variable for each protein. **E**. Untreated control osteosarcoma xenograft tumors and tumors harvested from mice treated with eribulin for 48 hours were lysed and assessed by immunoblot using antibodies against p27, STMN1, P-gp, p-MAPK and MAPK. GAPDH was loading control. **F**. Lysates of OS1 and OS9 xenograft tumors either untreated or treated with eribulin were incubated with anti-STMN1 antibody. Immunoblots of immunoprecipitated complexes were probed with antibodies against STMN1 and p27. The extent of coimmunoprecipitation is variable for each protein. **G**. Immunoblot of STMN1 protein following treatment of SaOS and **H**. 143B cells for 24 hours with siRNA targeting STMN1. STMN1 knockdown (siRNA STMN1) and STMN1 expressing cells (siRNA C) were treated with eribulin and cell viability was measured by cell titer blue assay. The percentage of viable cells for each group is shown relative to cells treated with control siRNA. Data are presented as mean absorbance ±SE of six replicates, n = 6.

Eribulin is also a substrate for the P-glycoprotein (P-gp) drug efflux pump and has decreased *in vitro* activity against cells overexpressing the P-gp [7]. Immunoblot analysis of P-gp in the xenograft tumors shown in Figure 4E, indicates that P-gp is highly expressed in OS9, OS17 and OS33 tumors, but the latter two are sensitive to the drug. Although P-gp likely alters the absorption, cytoplasmic concentration and excretion of eribulin by cells within these tumors, there was no correlation with drug sensitivity. Moreover, we examined the effect of eribulin on cell proliferative pathways. In agreement with *in vitro* findings, eribulin increased levels of p-MAPK in most tumors (Figure 4E), as observed in SaOS and 143B cell lines (Figure 1F). This indicates that activation of this cell proliferative pathway may be induced in response to microtubule targeting therapy, but is not unique to tumors that are resistant to therapy.

### Inducible βIII–tubulin correlates with lower sensitivity to eribulin in osteosarcoma cells and xenograft tumors

Overexpression of the βIII-tubulin isotype has been implicated as a marker of resistance to microtubule inhibitors, although this depends on tumor type and stage [30]. The resistant osteosarcoma xenograft tumors express low levels of *TUBB3* mRNA compared to HFL1 fibroblasts (Figure 5A). However, 48 hours after eribulin treatment, *TUBB3* mRNA expression was significantly upregulated in both of the resistant tumors (2.4 fold in OS9 and 2.9 fold in OS31, p = 0.05), and 1.6–fold in one of the sensitive tumors (OS33). With the exception of OS33, inducible *TUBB3* generally correlated with low eribulin activity (Figure 5B). In contrast, *TUBB3* mRNA levels decreased following eribulin treatment for OS1 and OS2 and no significant differences in *TUBB3* transcripts were observed between OS17 control and treated tumors (1.1-fold). βIII-tubulin expression was also determined in SaOS and 143B cell lines after eribulin treatment for 48 hours by real time RT-PCR and immunoblot. βIII-tubulin mRNA expression increased in both cell lines compared to controls (Figure 5C), corresponding increases in protein expression was observed in SaOS but not in 143B cells (Figure 5D). These results suggest that the specific induction of *TUBB3* may be of fundamental importance in the overall response to eribulin in osteosarcoma, and may have prognostic or predictive value in different settings and tumors.

**Figure 5:** βIII-tubulin expression in osteosarcoma cell lines and tumors **A**. Quantitative RT-PCR of *TUBB3* mRNA derived from SaOS, 143B and each osteosarcoma xenograft tumor, shown as –fold change relative to HFL1. **B**. Quantitative RT-PCR of *TUBB3* mRNA derived from untreated and eribulin-treated osteosarcoma xenograft tumors and **C**. SaOS and 143B cell lines. Data is shown as –fold change in treated tumors relative to untreated control tumors. **D**. Immunoblot of untreated, eribulin treated and washout (W/O) lysates of SaOS and 143B cells using antibodies against βIII-tubulin. GAPDH was loading control.

## DISCUSSION

Despite the development of several targeted therapies directed against cancer-specific pathways, cytotoxic treatments remain important clinical tools. Current efforts focus on using novel therapies targeting potential tumor vulnerabilities via genomic aberrations and biological pathways that support the malignant phenotype. A major question of clinical significance is whether tumors that show chromosome instability, such as osteosarcoma, are more or less sensitive to antimitotic drug-induced cell death. Historically, microtubule inhibitors have not had a prominent role in the treatment of osteosarcoma. Given the robust preclinical activity of microtubule inhibitors in the PPTP osteosarcoma panel, we investigated treatment effects on multiple processes that are sensitive to the loss of microtubule function.

This study confirmed the previously reported potency of eribulin in preclinical osteosarcoma models [11]. Here we demonstrate that eribulin disrupted microtubule networks in osteosarcoma cells and arrested cell cycle progression at mitosis, which caused mitotic catastrophe and subsequent cell death (Figure 6). MAPK, STAT3 and Akt are key effectors in three of the major signal transduction pathways through which growth factor signaling is mediated in osteosarcoma. The STAT3 and Akt signaling pathways were inhibited, indicating potent activity against the proliferation of cell lines and xenograft tumors. Nonetheless, the failure of eribulin to improve outcome in pediatric patients with recurrent osteosarcoma (AOST1322, NCT02097238) highlights current challenges for future opportunities in the development of eribulin therapies. In addition, in two recent, large-scale, randomized, phase 3 clinical studies of eribulin in patients with metastatic breast cancer, patients in the eribulin arm appeared to benefit more in terms of overall survival (OS) without corresponding increases in PFS [10, 31]. However, to date eribulin is the only single-agent that has been shown to prolong overall survival in patients with heavily pretreated metastatic breast cancer. Toxicity and pharmacokinetic evaluation of eribulin is not yet reported for pediatric patients. In adults with solid tumors, eribulin is primarily metabolized in the liver by the cytochrome P450 microenzyme CYP3A4, but does not increase levels of CYP3A4 substrates in blood plasma or microenzymes [32]. The drug is eliminated primarily unchanged in the feces (61%) and to a lesser degree in the urine (8%) [33]. These clinical outcomes warrant broader investigations of molecular and drug metabolism studies to provide comprehensive understanding why predicted mechanisms of tumor response to eribulin do not always translate into the anticipated clinical benefits for pediatric patients.

**Figure 6:** Summary of cellular response to eribulin in osteosarcoma A schematic depiction of mechanisms of cell death and cell proliferation in response to eribulin in osteosarcoma.

One overall concern regarding the translation of drugs targeting microtubules in preclinical models to clinical studies is that these agents cause cell death via mitotic arrest in rapidly dividing cells. The rationale for targeting cell proliferation stems from the assumption that tumors consist of more actively dividing cells than normal tissues. However, tumors grow slowly in humans when compared to tumors growing in preclinical animal or cell culture models. Thus the anti-tumor activity of these agents in humans is anticipated to be achieved more slowly than the rate seen *in vitro* in cell lines and *in vivo* in xenograft tumors grown in mice. In support of this theory, we have shown that while the initial responses of microtubule destabilization and mitotic arrest occur rapidly, both cell lines and tumors harbor a fraction of cells that remain viable at high concentrations of eribulin. We further show that proliferation of treated cells is restored following drug washout, confirming that mitotic arrest is reversible and cell cycle progression is restored upon drug removal. Though irreversible mitotic blockade by eribulin has been reported [34], our results are in agreement with other models that suggest some cells undergo mitotic slippage in the presence of antimitotic agents and remain viable [35, 36]. Further, these cells may exhibit aneuploidy arising from abnormal interphase nuclei. However, approximately 90% of solid tumors are aneuploid [36], and several osteosarcoma cell lines [37, 38] and tumors may have inherent mechanisms to adapt to errors due to faulty DNA replication [39].

Acquired drug resistance is also a major hurdle to the successful treatment of osteosarcoma. In general, osteosarcoma tumors can develop one or more acquired mechanisms of resistance with chemotherapy. Importantly, in the PPTP osteosarcoma xenograft models, tumor progression was reported for two tumors in response to eribulin therapy [11]. It is well known that the status of gene products, including p53, Bcl-2 and p21 contribute to resistance to the therapeutic induction of apoptosis [40]. Lack of apoptosis was confirmed *in vitro* in osteosarcoma cells that did not undergo Bcl-2 inhibition, or caspase-3 and PARP cleavage to initiate the signal transduction cascade leading to apoptotic cell death. Therefore, therapies that promote other types of cell death, such as programmed necrosis, may be useful in treating tumors with inherent aneuploidy such as osteosarcoma. Further validation of these compounds and optimization of their activity in the clinical setting will improve our ability to induce effective pro-apoptotic therapies in patients with osteosarcoma.

The β-tubulin subunit of the α/β-tubulin heterodimer is the cellular target of clinically used tubulin-binding agents. It is therefore anticipated that mechanisms of drug resistance could involve the differential expression of specific β-tubulin isotypes as well as microtubule-associated proteins (MAPs) and microtubule-interacting proteins (e.g. STMN1). The molecular functions of these protein changes in response to eribulin can influence the action of tubulin binding agents by modulating microtubule dynamics, drug binding and/or cell signaling. Given that eribulin does not disrupt STMN1 binding to p27 at low nanomolar concentrations *in vitro* and *in vivo*, we suggest the aberrant accumulation of STMN1/p27 complexes which do not bind unpolymerized tubulin are implicated in increases in the rate of mitosis through upregulation of microtubule stability [28]. These resistance mechanisms occurred in combination with specific overexpression of the βIII-tubulin isotype emphasizing that multiple, complex and likely interrelated mechanisms of drug response are involved in the overall response to eribulin, including P-gp mediated drug efflux. It is noteworthy, that treatment of human breast cancer cells with 60 nM eribulin for 4 hours attained intracellular concentrations of 3.5 μM in order to achieve mitotic arrest [21]. In contrast, drug washout resulted in complete loss of intracellular eribulin accumulation after 24 hours [21]. Our findings suggest that eribulin elicits stochastic toxicity but, that not all cells undergo mitotic catastrophe during the time of peak drug concentration. This indicates that drug effects are strongly dose-dependent. In the clinical administration of eribulin for metastatic breast cancer, a moderately intermittent dosing schedule is typically used (days 1 and 8 of a 21-day cycle) which is consistent with optimum preclinical effectiveness for osteosarcoma [7, 11]. This dosing regimen may not be appropriate for osteosarcoma patients and further dose-dependent studies are required to provide consistent anti-tumor activity with a better safety profile for pediatric patients. Other preclinical studies have suggested that eribulin may further alter tumor biology by processes independent of mitosis including remodeling the tumor vasculature, reversing features of epithelial-mesenchymal transitions and decreasing the migration and invasive capacity of tumor cells [18]. These additional effects may explain, at least in part, the clinical benefits of eribulin on OS than PFS or response rates observed in breast cancer patients.

In conclusion, we have demonstrated that the primary mechanism of action of eribulin in osteosarcoma is destabilization of microtubules, cell cycle arrest, mitotic catastrophe and cell death. We also show specific tumor-acquired responses to eribulin could lead to escape from mitotic arrest, causing cell proliferation and survival. Overexpression of critical proteins involved in microtubule dynamics including STMN1 and p27, and cyclin B1 in mitosis may serve as predictors to eribulin therapy. The development of such biomarkers may contribute to the understanding of eribulin activity in different tumors and facilitate the stratification of patients most likely to respond to treatment. These mechanistic studies are informative to the interpretation of current clinical observations and suggest that combining eribulin to disrupt microtubule dynamics with cytotoxic agents that induce DNA damage, may enhance osteosarcoma tumor responses by additive or synergistic modes of action. Drug combinations with adjunct agents that disrupt mitosis without affecting microtubules may also augment the effect of eribulin [41]. More in depth studies of tumor biology are deemed necessary to comprehensively unravel the complex tumor responses to eribulin, to develop safe and effective treatment strategies with broader activity and greater toxicities against pediatric osteosarcoma.

## MATERIALS AND METHODS

### Materials

Antibodies against Akt, p-Akt (Ser473), signal transducer and activator of transcription 3 (STAT3), p-STAT3 (Y705), mitogen-activated protein kinase (MAPK), p42/44-MAPK, cyclin B1, β-tubulin, *γ*-H2AX, PARP, cleaved PARP, caspase-3, Bcl-2, Receptor-interacting protein-1 (RIP1), stathmin-1 (STMN1), p27(Kip1) and GAPDH were purchased from Cell Signaling Technology (Danvers, MA). Eribulin mesylate (Halaven, Eisai Inc.) was purchased from the pharmacy at AIDHC and olesoxime was purchased from Sigma-Aldrich (St. Louis, MO).

### Osteosarcoma xenograft tumors and cell lines

The OS1, OS2, OS9, OS17, OS31, and OS33 tumor lines were generously provided by the Pediatric Preclinical Testing Program (Dr. Richard Gorlick, Albert Einstein College of Medicine, Bronx, NY). These lines are maintained by serial passage in severe combined immune deficient (SCID) mice as described previously by the Pediatric Preclinical Testing Program [12]. The human fibroblast cell line HFL1 (ATCC, Chicago, IL) was cultured in F-12K medium. Osteosarcoma cell lines SaOS and 143B were grown in McCoy's 5A and Minimum Essential Medium (MEM), respectively. Media were supplemented with 10% FBS and 1% penicillin/streptomycin. Cells were maintained at 37°C in a 5% CO2 incubator. All cell lines, media and supplements were obtained from the American Type Culture Collection (ATCC, Chicago, IL). Cells were maintained in 37°C incubators, in an atmosphere of 5% CO_2_ with 100% humidity.

### Drug treatment

SaOS and 143B cells were cultured in respective media (described above) overnight without drug then treated for 24, 48 or 72 hours with eribulin diluted in media without antibiotics and anti-mycotics (Invitrogen, CA). The term drug washout was used to describe pretreatment with concentrations of eribulin that were cytotoxic, followed by PBS washes and the addition of either drug-free medium or low dose eribulin (1 nM).

### Cell proliferation assay

The CellTiter-Blue Cell Viability Assay (Promega, Madison, WI) was used to measure cell viability. Cells were plated in 96-well tissue culture plates at a concentration of 2x10^3^ cells per well and grown for 24 hours. At approximately 70% confluency for SaOS and 50% for 143B, cells were treated with eribulin at 0.01 nM to 1000 nM for 72 hours. At the end of treatments, cell titer blue reagent was added to the medium, incubated at 37°C for 4 hours and absorbance readings taken at 584 nm on a Victor Plate Reader (Perkin Elmer, St. Louis, MO).

### Immunoblot

Cells and xenograft tumors were treated with eribulin for protein extraction and immunoblot analysis. Briefly, cells or tumors were lysed in RIPA buffer with Halt protease and phosphatase inhibitor cocktails (Thermo Fisher Scientific, Rockford, IL). Equal amounts (25 μg) of protein were separated by SDS–PAGE, and electrotransferred onto nitrocellulose membranes. These were incubated with primary antibodies followed by horseradish peroxidase-conjugated secondary antibody (Cell Signaling, Danvers, MA). Protein bands were visualized using chemiluminescence detection (GE Healthcare, PA). GAPDH antibody was the loading control.

### Quantitative real-time PCR

Total RNA from cells treated with eribulin was isolated using Trizol reagent (Invitrogen, CA). Synthesis of cDNA was performed using the High Capacity cDNA Reverse Transcription kit (Life Technologies, Grand Island, NY) with random hexamers. cDNA was amplified using gene-specific primers and amplified DNA was measured by ABI Prism 7000 Sequence Detection System (Applied Biosystems, Foster City, CA). Gene expression analysis was conducted by comparison of ΔΔCt values for each sample. PCR primers used are listed in Supplementary Table S1.

### Immunofluorescence

SaOS and 143B cells (2×10^4^) grown on glass coverslips (pre-coated with 0.01% w/v poly-L-lysine) in 24-well plates were treated with 10 nM eribulin. After 24 hours, cells were fixed with 4% paraformaldehyde, permeabilized using 2% Triton X-100 in PBS, and blocked with 5% horse serum. Cells were immunostained with anti-β-tubulin antibody followed by Alexa Fluor 488-conjugated anti-rabbit IgG (Thermo Fisher Scientific, Rockford, IL) and counterstained with Hoechst 33342 dye (Invitrogen, CA) at a 1:1,000 dilution of the stock solution (10 mg/ml), for 30 minutes at room temperature. The coverslips were mounted in SlowFade Gold Anti-Fade Reagent (Thermo Fisher Scientific, Rockford, IL). Phase-contrast images were obtained using a Leica DM IL microscope equipped with a DFC420 camera and Leica Application Suite Software (Leica Microsystems GmbH, Wetzlar, Germany). Fluorescence images were captured using a Leica TCS SP5 scanning confocal microscope (Leica Microsystems Inc., Buffalo Grove, IL) using the 63× oil objective.

### Cell cycle analysis

SaOS and 143B cells (1×10^6^) were incubated with or without 10 nM eribulin. Cell cycle progression was investigated by propidium iodide staining (Sigma) after 24 hours. Briefly, cells were trypsinized, washed with PBS and fixed with 70% ethanol for 30 mins at −20°C. Cells were then washed with PBS, pelleted and resuspended in 500 μl of PI/RNase solution for 15 min at room temperature. Cell cycle analysis was performed using the NovoCyte flow cytometer (ACEA Biosciences, San Diego, CA).

### Immunoprecipitation

Immunoprecipitation was performed using whole cell and tumor lysates (see *Immunoblot* above). 500 μg of protein lysate was precleared with Protein-G beads (Invitrogen, CA) then incubated with anti-STMN1 antibody overnight at 4°C. Antibody-protein complexes were conjugated to Protein-G beads for 2 hours at 4°C and precipitated by centrifugation. Immunoprecipitated complexes were washed with PBST (phosphate buffered-saline containing 0.3% Tween-80) and immunoblot was performed as described above.

### Mitochondrial membrane potential assay

Mitochondria membrane potential was measured using the Mitochondrial Membrane Potential Assay Kit (II), purchased from Cell Signaling Technology (Danvers, MA), according to manufacturer's protocol. Briefly, SaOS and 143B cells were grown in 6-cm cell culture dishes and treated with eribulin for 30 mins and 24 hours, with CCCP (carbonylcyanide 3-chlorophenylhydrazone) for 15 mins, and olesoxime and eribulin simultaneously for 24 hours. Following treatments live cells were harvested and TMRE accumulation was determined by flow cytometry (Accuri C6, BD Biosciences, CA).

### siRNA transfection

ON-TARGETplus SMARTpool human STMN1 siRNA and non-targeting, control siRNA were purchased from Dharmacon (Lafayette, CO) for the transient knockdown of STMN1. siRNA oligonucleotides were transfected in SaOS and 143B cells using the Lipofectamine RNAiMAX Transfection Reagent (Thermo Fisher Scientific, Rockford, IL) according to manufacturer's protocol.

### *In vivo* tumor growth inhibition

CB17SC scid −/− female mice (Taconic Farms, Germantown, NY), were used to propagate subcutaneously implanted osteosarcoma tumors, as previously described [12]. All mice were maintained under barrier conditions and experiments were conducted using protocols and conditions approved by the institutional animal care and use committee of the appropriate consortium member. Three mice were used in each control or treatment group. When the tumors grew to 5 – 6 mm in diameter, eribulin (1 mg/kg) or vehicle (PBS) was intravenously administrated. At 24 and 48 hours following treatment, cell and tumors were immediately harvested on ice and snap frozen for the preparation of RNA and protein lysates.

### Statistical analysis

Eribulin-treated vs control groups were analyzed by the Dunnett multiple comparisons test using two-sided approaches. Values of P<0.05 were considered as statistically significant. Statistical analyses were performed using GraphPad Prism version 5.04 (GraphPad Software, La Jolla, CA).

## SUPPLEMENTARY FIGURES AND TABLE


